# International Criminal Law Protection of Environmental Rights and Sentencing Based on Artificial Intelligence

**DOI:** 10.1155/2022/4064135

**Published:** 2022-05-31

**Authors:** Jiaxin Wu, Heyong Wang, Ning Sun, Hongwei Wang, Danila Tatarinov

**Affiliations:** ^1^Harbin Institute of Technology, Harbin 150001, China; ^2^Al-Farabi Kazakh National University, Almaty 050000, Kazakhstan

## Abstract

Environmental problem is an international problem that transcends national boundaries and develops into regional and global environmental pollution and ecological problems. Facing the increasing environmental pollution, the international community has successively formulated many relevant environmental pollution prevention laws, but the world situation is complicated after all, environmental problems still emerge endlessly, and the protection of environmental rights has become the consensus of the international community. Environmental right is an integral part of human rights, and protecting environmental right is the concrete expression and proper meaning of protecting human rights. Using international criminal law to protect environmental rights will play a positive role in global environmental protection. As with the development of computer technology, the research of machine learning has gradually transferred to the field of social science, especially the judicial field. While sentencing is a crucial part of environmental crime, this paper studies the sentencing of environmental rights cases from the perspective of international criminal law and uses Convolutional Neural Networks (CNN) to determine the sentencing of environmental rights cases. Through the experiment on the Integrated Database (IDB) dataset, the results show that the introduction of CNN improves the effect of the sentencing term prediction model and the fine prediction model significantly. The CNN-based model scored 91.6542 in the sentencing term prediction model and 90.8890 in the fine prediction model.

## 1. Introduction

International criminal law is generated and developed in the process of the international community fighting against international crimes, which is an important force in fighting international crime [1]. In recent years, there are two trends deserving attention in the development of international criminal law. On the one hand, the international community has continuously expanded and developed new fields of international cooperation in controlling international crime by concluding international criminal law conventions, stipulating new measures for controlling international crime, such as measures for controlling money laundering crime and measures for controlling corporate crime. On the other hand, these international criminal law conventions have begun to focus on the coordination between the basic principles of international law and specific rules, emphasizing that all states parties should abide by the basic principles of the Charter of the United Nations, such as “the sovereign equality of States” when performing their obligations under the conventions, and explicitly putting forward the provisions of “the protection of human rights” [2, 3]. Environmental right is an integral part of human rights. Therefore, protecting environmental right is an important task of human rights protection. International criminal law is the backbone of the fight against international crimes; it is generally believed that international criminal law should do something in the protection of environmental rights. Under the current international situation, it is the direction of environmental protection work to make full and reasonable use of international criminal law to protect environmental rights [4–6]. However, there are a few discussions on the protection of environmental rights in international criminal law.

Environmental right is generally defined internationally as the right to a good environment. However, this concept is in the process of being developed and there is no exact definition so far [7]. We believe that the environmental right is the right of harmonious coexistence between people and nature. Environmental problem is a social problem generated by modern capitalist mass production. Especially after World War II, with the economic development of major capitalist countries, environment and even environmental rights became an important topic of government policy. In Germany and the United States, environmental rights were discussed in the 1960s [8]. Environmental right was first defined by the Environmental Right Research Institute of Osaka Law Association of Japan as a pioneer of international environmental conference. It is believed that environmental right is the right to enjoy a good environment and control it [9]. In 1972, the United Nations held a conference on the Human Environment in Japan, and adopted the first principle of the Declaration on the Human Environment, which stipulates that everyone has the basic right to enjoy freedom, equality, and adequate living conditions in a good environment, and has the responsibility to protect and improve the environment for the present and future generations.

With the proposal and development of the environmental right theory, many countries and international organizations around the world have started relevant legislative activities. In the process of legislative practice, an inevitable problem is the division of environmental rights [10, 11]. We divide environmental rights into the following categories according to relevant environmental law theories: (1) Environmental rights of natural persons. Some scholars refer to a natural person's right to a healthy and living environment. (2) Environmental rights of legal persons and other organizations. It includes the legal right of legal persons and other organizations to utilize environmental resources and the right to discharge pollutants legally in the production process. (3) State environmental administrative power. Some scholars call this the national environmental right, which we do not think is appropriate because as the embodiment of public power, the state is mainly responsible for protecting natural resources and preventing air pollution, which is obviously a kind of power. We know that rights can be waived and that power cannot be “freely disposed of.” (4) Human environmental right. It refers to the right of good ecological environment that human beings as a whole should enjoy on the earth.

Although international environmental crime has not been comprehensively stipulated by international criminal law conventions, in view of the strong demand of the international community to bring violations of international environmental law into the international criminal system, international environmental crime as a major type of international crime is also a general trend, and how to its sentencing has become the focus of research [12]. In recent years, research progress on machine learning and deep learning in the field of natural science is in full swing. With the continuous development of computer technology, the research on machine learning has been gradually transferred to the field of social science, especially the judicial field. In traditional judicial judgments, the determination of sentencing often takes a lot of time and manpower, resulting in certain pressure on case trial judgments [13–15]. Therefore, the introduction of machine learning-assisted sentencing can effectively relieve this pressure, but the application of computer technology in the field of sentencing is not enough at present.

Our contributions are summarized as follows:

- We use convolutional neural networks (CNN) to determine the sentencing term and fine of environmental rights cases from the perspective of international criminal law.
- We analyze the protection of environmental rights under international criminal law.

The rest of this study is organized as follows.  Section 2 reviews related work. In Section 3, CNN-based sentencing term and fine research of environmental rights cases under international criminal law is presented. Experimental results and analysis are presented in Section 4.  Section 5 concludes this paper.

## 2. Related Work

Machine learning is the most common application of Artificial Intelligence (AI), which is the ability of computer systems to learn itself by analyzing large datasets and pattern recognition. Machine learning can draw conclusions and preprocess them based on probability, which is applicable to some data. In the long run, the application of AI in legal practice is unlimited, but currently it is commonly used in contract review, legal research, and results prediction. In [16], the author studied the relationship between AI technology and the rule of law, emphasizing that the rule of law was a mechanism of human prosperity. In [17], the author discussed the legal and rule-of-law assumptions and compared them with the assumptions of computing systems to illustrate the extent to which artificial legal intelligence provided responsible innovation in legal decision-making. In [18], the authors combined AI and deep learning algorithm in teaching design to enable students to carry out personalized learning tasks with pertinence, which was of great significance to cultivate high-level legal professionals. In [19], the author proposed to design and construct a data mining-based intelligent information acquisition system for cyber-economic crime using sensors and other technologies to realize the convergence of cyber-economic crime intelligence. In [20], the authors tried to establish a comprehensive scientific concept on the law of using AI in higher education and discuss the possibility of imposing civil sanctions on AI operations in the field of education.

Many strategies have been proposed for environmental right and sentencing. In [21], the author proposed a new type of norm integration and took human rights and environmental norms as examples to discuss the problem of norm integration. In [22], the author made a descriptive and normative economic analysis of international environmental rights. The link between environmental rights, environmental protection, and the courts has become increasingly prominent in recent years; in [23], the author attempted to determine the role of courts in efforts to protect the environment only on the basis of some case law. In [12], the authors studied the transformation from uncertain sentencing policy to decisive sentencing policy and the use of sentencing guidelines. In [24], the authors studied the role of sentencing guidance influence heuristics in shaping sentencing decisions through three methods. In [25], based on the data of hundreds of criminal cases in a county court in 2015, the authors studied the impact of legal and extrajudicial factors on sentencing results. In [26], the author presented some important problems on the different systems of sentencing procedures. In [27], the author studied the problem that using AI as an assisted system and machine learning algorithm might help suppress the sentencing difference between judges.

To the best of our knowledge, there is almost no application of AI to the protection of environmental rights from the perspective of international criminal law. In terms of sentencing, AI is not applied too. Therefore, based on AI, this paper studies the international criminal law protection of environmental rights and its corresponding sentencing issues.

## 3. CNN-Based Sentencing Term and Fine Research of Environmental Rights Cases under International Criminal Law

### 3.1. Basic Structure of the Model

This paper mainly considers the study of environmental rights cases in international criminal law and the term and fine in the sentencing system. Machine learning-assisted sentencing refers to predicting the specific value of term and fine in a given case through modeling under the condition of the fact text. Since it is difficult to find the factual case text of international criminal law protecting environmental rights, therefore, we use the Federal Court Cases Integrated Database (IDB) provided by the Federal Judicial Center for experiments. The IDB has case data of criminal, civil, appellate, and bankruptcy cases.

At first, data preprocessing is performed on the case text in IDB, and the English text is segmented by identifying space based on the case text data cleaning. Then, the text features of the case text data are analyzed, from which high-frequency words and low-frequency words are obtained. On this basis, the text data after word segmentation are cleaned and filtered, and the text word vectors are constructed based on Word2Vec. Finally, according to the word vector, the corresponding prediction model of sentencing and fine of environmental rights cases is constructed, the evaluation system of the model is constructed to evaluate the model according to the distribution characteristics of sentencing and fine, and some conclusions are obtained from the evaluation results of the model.

Generally, when using CNN for text analysis, the input layer inputs the text directly and then the embedding layer constructs the word vector. In this study, the basic CNN model has been modified slightly, and the embedding vector pre-trained by Word2Vec is input directly into the network. However, the application of Word2Vec in a CNN model is different from the averaging of all word segmentation in the machine learning model. It directly converts the text after word segmentation into a numerical matrix, i.e., each case text is expressed into a numerical matrix for later model building.

CNN is one of the most widely popular deep learning algorithms, and it can achieve a good learning effect on many tasks. CNN can use its unique structure to analyze the text and discover the hidden information in the text. Especially on the premise of large-scale data, CNN is more suitable for text analysis than traditional machine learning methods [28]. This paper attempts to build a sentencing prediction model and a fine prediction model through CNN.

Figure 1 shows the basic structure of CNN used in this paper in analyzing and processing the text of environmental rights cases. It is a two-dimensional word vector matrix of *k* × *n* obtained by the Word2Vec method at the input layer, where *k* represents the length of a case text composed of words *k*_1_, *k*_2_, *k*_3_,…, *k*_*i*_, and *n* represents the word vector dimension of each word. Afterwards, the collection and extraction of vector feature information are mainly carried out in the convolutional and pooling layers, and then the features extracted in the previous steps are output through the fully connected layer. Finally, the prediction effect of the model can be obtained through the output layer. In this way, the corresponding model of CNN for predicting sentencing and fine is built.

### 3.2. Framework for the Model

On the basis of the schematic diagram shown in Figure 1, the functions of each layer in CNN and the specific method in this paper are introduced emphatically.

#### 3.2.1. Input Layer

In this paper, the input of CNN is the word vector matrix processed by Word2Vec, and the output is the sentencing and fine of each environmental rights case. Before constructing the word vector, it is necessary to process the dataset filtered by word segmentation. In the IDB dataset, 20000 words are reserved after word segmentation. Considering that each text has a large length gap after word segmentation, the text length is limited to 400. Text length with less than 400 is supplemented with 0, and text length with more than 400 is truncated. After fixing the length of each text to 400, the environmental rights case text after segmentation needs to be transformed into a vector representation. The dimension of word vector in Word2Vec is set as 400. Since each row in the matrix represents a word participle, the case after each word segmentation becomes a matrix of 400 *∗* 400, and then the vector matrix is input into the network for training.

#### 3.2.2. Convolutional Layer

It can be seen from the operation of the input layer that the environmental right case text is input in the convolutional layer in the form of a two-dimensional matrix, and the feature information in the case text can be extracted by the convolution operation in the convolutional layer. In addition, in convolution operation, the selection of an activation function is also very important. In this paper, the Rectified Linear Function (ReLU) function that can accelerate the convergence speed in training the case text word vector data is selected.

#### 3.2.3. Pooling Layer

After obtaining the text features of environmental right cases through convolution operation, if these features are directly used for the regression prediction of sentencing, the calculation amount will be too large due to the large amount of feature data, and the training process will be relatively slow. On the premise of fully retaining useful features, to simplify the number of parameters of CNN and reduce the computational complexity, it is necessary to compress and merge the features of case texts with similar semantics in the pooling layer, which is equivalent to extracting features again and filtering some useless features to meet the requirement of reducing the number of parameters in the model. Common pooling methods are average pooling, maximum pooling, and random pooling, and maximum pooling is used to preserve more features.

#### 3.2.4. Fully Connected Layer and Output Layer

The pooling structures are aggregated in the fully connected layer. In Keras, the connections between neurons in the fully connected layer are dense, and this layer is defined as the Dense layer in order to represent this relationship [29]. We define the fully connected layer through the Dense function to obtain the final feature vector of environmental rights case text, which is input into the final output layer to obtain the final prediction results of the sentencing term and fine.

## 4. Experiment and Results Analysis

### 4.1. Parameters' Setting

In the construction of CNN, parameters involved in the model need to be set through analysis, including the text length of the environment right case text input to the CNN, the size of the dictionary constructed by the case text, the dimension of the word vector, the size of the convolution kernel of the CNN, the value of the Dropout parameter, and the number of iterations of training CNN.

Earlier in the paper, it has been known that the length of text of environmental rights cases should be set to 400 in terms of sentencing and fine prediction. In the IDB dataset, 20000 words are reserved after word segmentation. For other parameter settings, generally speaking, the more dimensions of word vector constructed by the case text, the better the prediction effect of the corresponding model. However, if the word vector dimension continues to increase, the complexity of the network structure will also continue to increase, which will bring a lot of calculations, greatly extend the training time of the model, resulting in the reliability of the prediction effect being decreased. The smaller the size of the convolution kernel, the less parameters and computation are needed to train the CNN. Therefore, the minimum convolution kernel size should be selected on the premise that the prediction effect can be guaranteed. Generally, a smaller convolution kernel size with a slightly larger number of convolution kernels is recommended with the support of computer performance. When the sample size is large, it can be considered to reduce the value of the batch size. However, if the sample size is blindly reduced, it is likely to be non-convergence. Therefore, selecting an appropriate batch size value is helpful to improve the efficiency of model operation.

The settings of parameters in sentencing term and fine prediction of CNN in this paper are shown in Table 1.

### 4.2. Results' Analysis

In traditional regression prediction, most of the evaluation metrics consider using mean square error. Due to the particularity of sentencing and fine prediction, to make the model results more clear, we try to score the model results, and the score results can also be used for the comparison between models in the later stage. The mean absolute error after transformation considers the distance *d*_*i*_ between the predicted value and the true value after sample *x*_*i*_ processing. The larger the *d*_*i*_, the larger the distance between the predicted value and the real value, and the farther the predicted value is from the real situation, the worse the prediction effect of the model. Therefore, *d*_*i*_ is used to construct the evaluation metric of the machine learning-assisted sentencing model, i.e., the score of the model. The model can be evaluated according to the score of the model.

(1) $$\begin{array}{c} d_{i}=\log\left(y_{i}^{\prime }+1\right)-\log\left(y_{i}+1\right), \end{array}$$

where *y*_*i*_′ is the predicted value of sample *x*_*i*_, and *y*_*i*_ is the true value of sample *x*_*i*_.

The model score *s* is defined as follows:

(2) $$\begin{array}{c} s=\sum_{i=1}^{n}s_{i}\left\{\begin{array}{cc} s_{i}=1, & d_{i}\leq 0.2,\\ s_{i}=0.8, & 0.2<d_{i}\leq 0.4,\\ s_{i}=0.6, & 0.4<d_{i}\leq 0.6,\\ s_{i}=0.4, & 0.6<d_{i}\leq 0.8,\\ s_{i}=0.2, & 0.8<d_{i}\leq 1,\\ s_{i}=0, & d_{i}>1. \end{array}\right) \end{array}$$

#### 4.2.1. Results for Sentencing Term Prediction

In terms of sentencing term prediction, the CNN is built to predict the sentencing term in environmental rights cases protected by international criminal law. At the same time, three traditional machine learning methods such as random forest (RF) [30], artificial neural network (ANN) [31], and eXtreme Gradient Boosting (XGBoost) models [32] also tried to predict the sentencing term. On the basis of the prediction results, the above constructed scoring system is used to evaluate and compare each method.  Table 2 shows the scores of sentencing term prediction in the training set and test set under the four methods. It can be seen that in the traditional machine learning model, RF performs worse on the training set and test set compared with the other two methods, and the score is lower, while the XGBoost model has the highest score. However, regardless of whether it is RF, ANN, or XGBoost, the model scores are actually low. After using the CNN method, the model scores on the training set and test set have been significantly improved. It can be considered that compared with traditional machine learning methods, CNN is more effective in predicting the sentencing term of environmental rights cases.

#### 4.2.2. Results for Fine Prediction

The CNN model is built with the IDB dataset for the prediction of fine, and RF, ANN, and XGBoost models also tried, respectively. The constructed scoring system is used for evaluation and comparison, and the results are shown in Table 3. It can be seen that the fine prediction model has basically the same effect as the sentencing term prediction model in the traditional machine learning model. The CNN model also has the highest score, while the RF model has the lowest score. The CNN greatly improves the model scores for both the sentencing term prediction model and the fine prediction model, but the model scores on the fine are lower than that of the sentencing term.

In terms of feature extraction, every dimension of word vectors is trained as a feature in the traditional machine learning-assisted sentencing model. However, the CNN adopted in this paper can automatically extract feature information of the case text, which can save time and effort. Moreover, the features automatically extracted have stronger discriminant ability for later analysis. At the same time, when CNN is used to model and predict the environmental rights cases, the feature extraction and results prediction are performed in the CNN as a whole, which can maximize the performance of feature extraction and model prediction.

#### 4.2.3. Imbalance of Sentencing in International Criminal Law

When we understand and determine the scope of sentencing circumstances, we can consider the weight of each circumstance in sentencing. The proportion of different sentencing circumstances in sentencing has not yet formed a unified provision in the international criminal court. However, according to the handling of relevant cases, we can know that the role of bad physical condition and confession in sentencing cannot be underestimated, but it is always difficult to judge the proportion of many factors in the final sentencing. In this case, in order to clearly inform the aggravation or reduction of criminal law and avoid paying too much attention to sentencing factors as much as possible, the proportion of sentencing circumstances must be determined.

It should be noted that this proportion cannot be accurately determined to a number, only for its relevant provisions and requirements. In determining the proportion of sentencing circumstances, the purpose of punishment should be considered. For international criminal law, it is necessary to always adhere to the purpose of retribution and pay necessary attention to the special purpose of prevention. Therefore, the two purposes of sentencing should be determined in combination with the proportion of circumstances. However, it is impossible to cover all sentencing circumstances, which can only be determined at the general level. Hence, in the determination of sentencing circumstances, the following aspects should be followed: (i) The determination of circumstances of sentencing should be related to the purpose of criminal law. (ii) If it is an aggravating circumstance, because it will directly increase the penalty and cause serious damage to the rights of the defendant, it should be restricted according to the explicit provisions, and the analogy is not allowed to exist. At the same time, aggravating circumstances only include the scope of the implementation of the crime and the cause of a close relationship between the criminal act and the offender. In addition, the requirements for mitigating circumstances need not be too strict, and the scope should be appropriately expanded. As long as there is no direct connection with the criminal act, it can be regarded as the reason for mitigating the circumstances of punishment. (iii) No double evaluation is allowed. Specifically, for the same reasons of the case, the penalty should not be evaluated repeatedly, so as to effectively avoid the excessive increase or reduction of the defendant's punishment.

When determining the proportion of sentencing circumstances, on the one hand, the determination of international criminal law to punish international criminal acts should be shown, so it is not allowed to focus on the sentencing circumstances for preventive purposes. On the other hand, if the increase or decrease of the proportion of criminal law for no less than one circumstance exceeds the scope of the established proportion, specific reasons must be elaborated in detail.

For international criminal law, the criminal law itself is in the initial stage of development, and thus the problem of sentencing imbalance has not received necessary attention. That is to say, theoretical research related to sentencing imbalance is not mature, and there is no effective system to overcome it in practice. Therefore, we must attach great importance to the study of sentencing imbalance from the perspective of international criminal law.

#### 4.2.4. International Criminal Law Protection of Environmental Rights

Given the above, we analyze the environmental rights sentencing under the protection of international criminal law assisted by machine learning. However, there are more and more provisions in international environmental crime in international treaties, and the theory and practice of using international criminal law to protect environmental rights are becoming more and more mature. Then, as a relatively independent international criminal law norm, we try to analyze what constitutive elements of international environmental crime should include.

1. Object of international environmental crime. The object violated by principal crime is the ecological environment (resources) on which human beings depend, including environmental elements such as atmosphere, water, ocean, forest, grassland, and flora and fauna. In the case of pollution in outer space, it should be considered an international environmental crime if it violates the provisions of relevant international conventions.
2. Subject of international environmental crime. The subjects of international environmental crime include natural persons, legal persons, and other organizations and countries, but there is a great controversy on whether a country accepts criminal responsibility for international environmental crime. We believe that with the continuous improvement of international criminal law legislation and international theory of environmental crime, incorporating the country into the subject of international environmental crime fits the needs of current international environmental protection work. Apparently, the way in which a country assumes criminal responsibility for international environmental crime is not clearly defined in the existing documents such as international criminal law. Therefore, theoretical perfection and system innovation are urgently required in future research. At present, it has gradually been accepted by the international community to include the country as the subject of international environmental crime.
3. Objective aspects of international environmental crime. Principal crime is objectively manifested as a violation of the prohibitive provisions of international criminal law, a serious damage to human ecological environment, and a harmful act subject to international criminal responsibility. According to the different behavior modes, harmful behaviors can be divided into actions and omissions. According to the different behavioral means, harmful behaviors can be divided into those that destroy natural resources and those that pollute the environment. If there are specific classifications of harmful behaviors, they can be roughly divided into the following categories: (i) Air pollution; (ii) Marine pollution; (iii) Outer space pollution, such as the test and use of nuclear weapons and weapons of mass destruction; and (iv) Transfer of pollution.
4. Subjective aspects of international environmental crime. The subjective aspect of international environmental crime can be intentional or negligent. Although some scholars disapprove of negligence as the subjective element of the crime, we believe it is against the efforts of the international community to strengthen environmental protection. Generally, the destruction of natural resources is mostly intentional while the pollution of the environment is mostly negligent.

## 5. Conclusions

International criminal law plays an irreplaceable role in the protection of environmental rights. Using international criminal law to protect environmental rights is consistent with the current general promotion of human rights. In this paper, CNN is used to study the sentencing of environmental rights from the perspective of international criminal law, including the prediction of the sentencing term and fine. The corresponding sentencing term or fine is obtained through the description of environmental rights case text. To make the prediction effect of the sentencing term or fine more clearly displayed, the distance between the predicted sentencing term or fine and the true value is considered to construct the score; thus, the evaluation and analysis of the predicting effect of the model can be realized, and the reference basis can be provided for the selection of different assisted sentencing models. The experimental results show that the CNN-based model achieves good prediction effect on the test set. In the computer-assisted sentencing of environmental crime, besides the influence of criminal circumstances on the results of sentencing, there are other impact factors such as charges, judges, regions, etc. We should fully consider all possible factors that may affect the results of sentencing, and adopt more complex machine learning models or integrate more knowledge models to build more effective models, so that computer-assisted sentencing can be more effectively used in the actual case trial.

## Figures and Tables

**Figure 1:** CNN structure diagram.

**Table 1:** Parameter settings for CNN.

Parameter	Setting
Size of text	400
Embedding word vector dimension	400
Size of kernel	3
Number of kernels	512
Batch size	256
Dropout rate	0.1

**Table 2:** Sentencing term prediction model score.

	RF	ANN	XGBoost	CNN
Score of training set	64.5917	66.3994	67.4135	93.3621
Score of test set	58.6248	61.2346	62.3448	91.6542

**Table 3:** Fine prediction model score.

	RF	ANN	XGBoost	CNN
Score of training set	62.7463	65.3524	67.0012	92.4256
Score of test set	56.2615	60.7631	60.0237	90.8890

## Data Availability

All data used to support the findings of the study are included within this paper.

## References

[1] Rapp K. (2020). Law and contestation in international negotiations. *Review of International Studies*.

[2] Christensen M. J. (2019). The judiciary of international criminal law. *Journal of International Criminal Justice*.

[3] Redwood H., Goozee H. (2021). Shifting accounts of justice: the legalisation and politicisation of international criminal justice. *Social & Legal Studies*.

[4] Killean R. (2021). From ecocide to eco-sensitivity: “greening” reparations at the international criminal court. *International Journal of Human Rights*.

[5] Gellers J. C., Jeffords C. (2018). Toward environmental democracy? procedural environmental rights and environmental justice. *Global Environmental Politics*.

[6] Xu Y., Huang X., Bao H. X. H. (2018). Rural land rights reform and agro-environmental sustainability: empirical evidence from China. *Land Use Policy*.

[7] Gibert K., Horsburgh J. S., Athanasiadis I. N., Holmes G. (2018). Environmental data science. *Environmental Modelling & Software*.

[8] Ponce P., Khan S. A. R. (2021). A causal link between renewable energy, energy efficiency, property rights, and CO_2_ emissions in developed countries: a road map for environmental sustainability. *Environmental Science and Pollution Research*.

[9] Hubert A. M. (2020). The human right to science and its relationship to international environmental law. *European Journal of International Law*.

[10] Scotford E. (2021). Legislation and the stress of environmental problems. *Current Legal Problems*.

[11] Brandi C., Blümer D., Morin J. F. (2019). When do international treaties matter for domestic environmental legislation?. *Global Environmental Politics*.

[12] Arazan C. L., Bales W. D., Blomberg T. G. (2019). Courtroom context and sentencing. *American Journal of Criminal Justice*.

[13] Li J., Zhang G., Yu L., Meng T. (2019). Research and design on cognitive computing framework for predicting judicial decisions. *Journal of Signal Processing Systems*.

[14] Medvedeva M., Vols M., Wieling M. (2020). Using machine learning to predict decisions of the European court of human rights. *Artificial Intelligence and Law*.

[15] Nowacki J. S. (2017). An intersectional approach to race/ethnicity, sex, and age disparity in federal sentencing outcomes: an examination of policy across time periods. *Criminology and Criminal Justice*.

[16] Greenstein S. (2021). Preserving the rule of law in the era of artificial intelligence (AI). *Artificial Intelligence and Law*.

[17] Hildebrandt M. (2018). Law as computation in the era of artificial legal intelligence: speaking law to the power of statistics. *University of Toronto Law Journal*.

[18] Xuan D., Zhu D., Xu W. (2021). The teaching pattern of law majors using artificial intelligence and deep neural network under educational psychology. *Frontiers in Psychology*.

[19] Tan T. (2021). Intelligent application of artificial intelligence internet of things technology in the economic and legal fields. *Mobile Information Systems*.

[20] Makarov T. G., Arslanov K. M., Kobchikova E. V., Opyhtina E. G., Barabanova S. V. (2022). Legal aspects of using artificial intelligence in higher education. *Mobility for Smart Cities and Regional Development—Challenges for Higher Education*.

[21] Gonenc D. (2021). Conceptualizing norm fusion through environmental rights. *Environmental Politics*.

[22] Reynolds J. L. (2019). An economic analysis of international environmental rights. *International Environmental Agreements: Politics, Law and Economics*.

[23] Soyapi C. B. (2020). A multijurisdictional assessment of the judiciary’s role in advancing environmental protection in Africa. *Hague Journal on The Rule of Law*.

[24] Marder I. D., Pina-Sanchez J. (2020). Nudge the judge? theorizing the interaction between heuristics, sentencing guidelines and sentence clustering. *Criminology and Criminal Justice*.

[25] Lin X., Liu S., Li E., Ma Y. (2021). Sentencing disparity and sentencing guidelines: the case of China. *Asian Journal of Criminology*.

[26] Plesnicar M. M. (2018). Sentencing procedures. *Revija za Kriminalistiko in Kriminologijo*.

[27] Ryberg J. (2021). Sentencing disparity and artificial intelligence. *The Journal of Value Inquiry*.

[28] Abas A. R., Elhenawy I., Zidan M., Othman M., Bert C. (2022). A deep learning model for detecting emotions from text. *CMC-Computers Materials & Continua*.

[29] Grattarola D., Alippi C. (2021). Graph neural networks in tensorflow and keras with spektral [application notes]. *IEEE Computational Intelligence Magazine*.

[30] Bai J., Li Y., Li J., Yang X., Jiang Y., Xia S. T. (2022). Multinomial random forest. *Pattern Recognition*.

[31] Fatima S. A., Ramli N., Taqvi S. A. A., Zabiri H. (2021). Prediction of industrial debutanizer column compositions using data-driven ANFIS- and ANN-based approaches. *Neural Computing & Applications*.

[32] Asselman A., Khaldi M., Aammou S. (2021). Enhancing the prediction of student performance based on the machine learning XGboost algorithm. *Interactive Learning Environments*.

